This article has been retracted.

# Systematic study of cilostazol on secondary stroke prevention: a meta-analysis

**DOI:** 10.1186/2047-783X-18-53

**Published:** 2013-12-06

**Authors:** Yining Qian, Qi Bi

**Affiliations:** 1 Department of Neurology, Beijing Anzhen Hospital, Capital Medical University, Beijing 100029, China

**Keywords:** Cilostazol, Ischemic stroke, Systematic reviews

## Abstract

**Background:**

To study the efficacy and safety of cilostazol on ischemic stroke prevention and treatment, systematic reviews of related clinical randomized controlled trials were analyzed.

**Methods:**

We searched the main databases for eligible trials including literature from January 1966 to November 2012 in MEDLINE, reports from 1980 to November 2012 in EMBASE, and all the studies published in EBSCO, Springer, Ovid, and Cochrane library citations. We also searched for keywords, including cilostazol and aspirin. RewMan 5.0 software was used to conduct the meta-analysis.

**Results:**

Our search yielded five eligible trials. The effects of cilostazol and aspirin on ischemic stroke prevention and treatment were almost equal (combined odds ratio (OR) 0.78, 95% confidence interval (CI) (0.59, 1.04)). Additionally, both magnetic resonance angiography (MRA) and transcranial Doppler (TCD) examination showed that cilostazol could significantly decrease the incidence of intracranial artery stenosis exacerbation (MRA: combined OR 0.22, 95% CI (0.07, 0.68); TCD: combined OR 0.17, 95% CI (0.05, 0.51)). In terms of adverse reactions, there were slightly fewer incidences of major bleeding with cilostazol than with aspirin (combined OR 0.38, 95% CI (0.24, 0.60)), and there was no difference in the number of heart palpitations between cilostazol and aspirin. However, the incidence of gastrointestinal disorders, dizziness, and headaches caused by cilostazol was greater.

**Conclusions:**

Cilostazol might be a more effective and safer alternative to aspirin for patients with ischemic stroke. Further studies are required to confirm whether cilostazol is a suitable therapeutic option for secondary stroke prevention in larger cohorts of patients with ischemic stroke.

## Background

Ischemic stroke, which indicated that ischemia is caused by blockage, is a major cause of death and disability worldwide, and contributes significant financial burdens [1]. Owing to this severe cost of ischemic stroke, secondary prevention, namely preclinical prevention, plays an important role in reducing mortality and morbidity [2]. Antiplatelet treatment is a mainstay in acute and long-term secondary stroke prevention [3]. The most widely used antiplatelet drug for stroke prevention is aspirin, which significantly reduces the recurrence rate of ischemic stroke [4]. However, the clinical application of aspirin is limited due to major hemorrhagic adverse effects. Although several studies concluded that the advantages of aspirin are enough to outweigh the risk of hemorrhagic infarctions in most populations [5], the potential of adverse effects for the application of aspirin still cannot be ignored, particularly for individuals in Asia [6]. Moreover, many studies also found that despite regular antiplatelet treatment, some patients experienced thromboembolic events [7-9]. Those patients are clinically designated as aspirin resistant or non-responders. The incidence of low response or non-response to aspirin ranges between 5% and 60% [9]. Therefore, searching for antiplatelet agents with minimum complications and drug resistant is important.

Cilostazol has been shown to be an alternative to aspirin for secondary prevention in patients with non-cardioembolic ischemic stroke [10]. Cilostazol is a selective phosphodiesterase 3 (PDE3) inhibitor, possessing a potentially powerful means to produce various pleiotropic effects. Currently, promoting evidence shows that cilostazol can serve as an antiplatelet agent. The effects of cilostazol on stroke prevention are caused by its protective effect against secondary cerebral infarctions [11]. Although cilostazol is widely used for the treatment of intermittent claudication with peripheral artery occlusion and for the prevention of ischemic stroke [12], reported clinical outcomes on its efficacy and side effects are conflicting, and systemic reviews are needed. In our paper, we assess the safety and efficacy of cilostazol versus aspirin for secondary stroke prevention in current clinical randomized controlled trials, aiming to provide guidance for their clinical application.

## Methods

### Search strategies

#### Research strategies

We fully researched MEDLINE, EMBASE, EBSCO, Springer, Ovid, and Cochrane library citations.

1) MEDLINE: January 1966 to November 2012, including established searches using a Cochrane Randomized Controlled Trials filter to identify randomized controlled trials combined with terms that will include cilostazol and aspirin.

2) EMBASE: 1980 to November 2012.

3) The Cochrane Central Register of Controlled Trials.

4) All reference lists of identified studies in EBSCO, Springer, Ovid, and Cochrane library citations.

#### Inclusion criteria

The published studies should be randomized controlled trials (RCTs), in which the patients were randomly grouped and accepted different interventions for comparison. All patients in the studies should have a medical history of ischemic stroke or transient ischemic attack and meet WHO criteria [13]. Patients should be older than 18 years. Therapeutic effects studied should include the incidence of ischemic stroke, the state of exacerbation of intracranial artery stenosis, and changes to the intima-media thickness. The following side effects should be noted: major bleeding, including intracranial hemorrhage and massive hemorrhage needing hospital blood transfusion, palpitation, gastrointestinal disorders (diarrhea, constipation, and so on), headaches, and dizziness.

Exclusion criteria are non-RCTs, patients with a history of gastrointestinal bleeding, bloody urine, conjunctival hemorrhageor patients with serious diseases, such as malignant neoplasm, heart failure, or renal failure.

### Quality assessment and data extraction

Quality assessment included the adequacy of the random allocation method, the hidden nature of the random allocation method, the adoption of blinding methods, and evaluation of withdrawals.

Extracted data included: (1) general information: such as the topic of research, authors, the sources of literatures and so on; (2) research characteristics: design scheme, research strategies, implementation methods, measures to prevent bias, main test results and so on; (3) outcome measures: such as follow-up time, treatment of data from patients lost to follow-up or withdrawing from the study, curative effects and side effects, collection of headcounts of each group and the number of various events.

### Statistical analysis

Meta-analysis was carried out by RevMan 5.0 provided by the Cochrane Collaboration. Odds ratios (OR) were used to determine effect size, along with 95% confidence interval (CI). Heterogeneity in results across studies was examined using the chi-square or tau- squaretest. When heterogeneity was not observed (*P* > 0.01,*I*^2^ ≤ 56%), the effect size was calculated based on a fixed-effects model; otherwise a random-effects model was used. The overall effect estimate was analyzed by Mantel-Haenszel method. All efficacy index analysis followed the principle of intentional analysis.

## Results

### Eligible trials

Using this retrieval method, five eligible trials published between 2005 and 2011 were found [14-18], containing 4,052 cases of patients from different countries including Japan, Korea, and China. Among the five eligible trials, four compared the efficacy of cilostazol and aspirin [14-17], and one compared cilostazol and a placebo based on aspirin usage [18]. With respect to main curative effects, four analyzed the incidence of ischemic stroke [14-17], and two analyzed exacerbation of intracranial artery stenosis [16,18], but no RCTs referred to intima-media thickness in carotid arteries of stroke patients. Regarding side effects, four analyzed major bleeding, dizziness and headaches [14-17], three analyzed palpitation [14,15,17], and three analyzed gastrointestinal disorders [14-16]. All five trials applied a random and double-blind method, but only one used allocation concealment [15].

### Efficacy analysis

#### Incidence of ischemic stroke

Four trials [14-17] compared the incidence of ischemic stroke in cilostazol groups and aspirin groups. A fixed-effects model was chosen, because of the poor heterogeneity (*P* = 0.77, *I*^2^ = 0%). The combined OR was 0.78 and 95% CI (0.59, 1.04), with no statistical significance (*Z* = 1.68, *P* = 0.09). Therefore, no difference was observed between cilostazol and aspirin groups in prevention and cure of ischemic stroke (see Figure 1).

**Figure 1:** **Forest plots of comparison of the incidence of ischemic stroke between cilostazol and aspirin groups in prevention and cure of ischemic stroke.** Heterogeneity test, chi-square statistic with degrees of freedom and *P* value; inconsistency among results, *I*^2^ test for overall effect, *Z* statistic with *P*. CI, confidence interval; df, degrees of freedom; M-H, Mantel-Haenszel method.

### Progression of intracranial artery stenosis

Two studies [16,18] focused on the progression of intracranial artery stenosis, with placebo and aspirin as the control, respectively. Magnetic resonance angiography (MRA) and transcranial Doppler (TCD) were applied in both studies to examine arteriostenosis. There was no heterogeneity in the results of MRA examination among studies (*P* = 0.25, *I*^2^ = 23%), and a fixed-effects model was adopted. The combined OR was 0.22 with 95% CI (0.07, 0.68), with statistical significance (*Z* = 2.63, *P* = 0.009). Therefore, according to MRA examination, cilostazol was more effective than aspirin in preventing intracranial artery stenosis progression (see Figure 2).

**Figure 2:** **Forest plots of comparison of the progression of intracranial artery stenosis (by magnetic resonance angiography) between cilostazol and aspirin groups in prevention and cure of ischemic stroke.** Heterogeneity test, chi-square statistic with degrees of freedom and *P* value; inconsistency among results, *I*^2^ test for overall effect, Z statistic with *P* value. CI, confidence interval; df, degrees of freedom; M-H, Mantel-Haenszel method.

No heterogeneity was observed in results of TCD examination among studies (*P* = 0.16, *I*^2^ = 50%), and a fixed-effects model was applied. The combined OR was 0.17 with 95% CI (0.05, 0.51), with statistical significance (*Z* = 3.12, *P* = 0.002). Therefore, according to TCD examination, cilostazol was superior to the control in prevention and treatment of intracranial artery stenosis progression (see Figure 3).

**Figure 3:** **Forest plots of the comparison of the exacerbation of intracranial artery stenosis (by transcranial Doppler) between cilostazol and aspirin group.** Heterogeneity test, chi-square statistic with degrees of freedom and *P* value; inconsistency among results, *I*^2^ test for overall effect, *Z* statistic with *P* value. CI, confidence interval; df, degrees of freedom; M-H, Mantel-Haenszel method.

### Adverse effects analysis

#### Major bleeding

Four eligible studies [14-17] compared the incidence of major bleeding in cilostazol and aspirin groups. Since no heterogeneity was observed (*P* = 0.93, *I*^2^ = 0%), a fixed-effects model was chosen. The combined OR was 0.38 and 95% CI (0.24, 0.60), with statistical significance (*Z* = 4.15, *P* < 0.0001). Thus, the incidence of major bleeding was slightly reduced with cilostazol, compared with aspirin (see Figure 4).

**Figure 4:** **Forest plots of the comparison of major bleeding between cilostazol and aspirin group.** Heterogeneity test, chi-squarestatistic with degrees of freedom and *P* value; inconsistency among results, *I*^2^ test for overall effect, *Z* statistic with *P* value. CI, confidence interval; df, degrees of freedom; M-H, Mantel-Haenszel method.

### Palpitation

Three trials [14,15,17] compared the incidence of palpitation in cilostazol and aspirin groups. A random-effects model was used for the heterogeneity (*P* < 0.01, *I*^2^ = 94%). The combined OR was 0.96 with 95% CI (0.15, 6.21), with no statistical significance (*Z* = 0.04, *P* = 0.97). So there was no difference in the side effect of heart palpitations between cilostazol and aspirin (see Figure 5).

**Figure 5:** **Forest plots of the comparison of palpitation between cilostazol and aspirin group.** Heterogeneity test, chi-squared statistic with degrees of freedom and *P* value; inconsistency among results, *I*^2^ test for overall effect, *Z* statistic with *P* value. CI, confidence interval; df: degrees of freedom, M-H, Mantel-Haenszel method.

### Gastrointestinal disorders

Three trials [14-16] compared the incidence of gastrointestinal disorders in cilostazol and aspirin groups. A fixed-effects model was used for the poor heterogeneity (*P* = 0.61, *I*^2^ = 0%). The combined OR was 1.23 with 95% CI (1.04, 1.46), with statistical significance (*Z* = 2.40, *P* = 0.02) (see Figure 6). Thus, the incidence of gastrointestinal disorders caused by cilostazol was higher than the incidence of gastrointestinal disorders caused by aspirin.

**Figure 6:** **Forest plots of the comparison of gastrointestinal disorders between cilostazol and aspirin group.** Heterogeneity test, chi-squarestatistic with degrees of freedom and *P* value; inconsistency among results, *I*^2^ test for overall effect, *Z* statistic with *P* value. CI, confidence interval; df, degrees of freedom; M-H, Mantel-Haenszel method.

### Dizziness

Four studies [14-17] compared the incidence of dizziness in cilostazol and aspirin groups. Fixed-effects model was used for the poor heterogeneity (*P* = 0.58, *I*^2^ = 0%). The combined OR was 1.44 with 95% CI (1.15, 1.80), with statistical significance (*Z* = 3.18, *P* = 0.001). Therefore, there was more dizziness associated with cilostazol than with aspirin (see Figure 7).

**Figure 7:** **Forest plots of the comparison of the incidence of dizziness between cilostazol and aspirin group.** Heterogeneity test, chi-squarestatistic with degrees of freedom and *P* value; inconsistency among results, *I*^2^ test for overall effect, *Z* statistic with *P* value.CI, confidence interval; df, degrees of freedom; M-H, Mantel-Haenszel method.

### Headache

Four studies [14-17] compared the incidence of headache in cilostazol and aspirin groups. A fixed-effects model was used for the poor heterogeneity (*P* = 0.09, *I*^2^ = 55%). The combined OR was 1.78 with 95% CI (1.52, 2.10), with statistical significance (*Z* = 6.97, *P* < 0.00001). Therefore, the prevalence of headaches with cilostazol was higher than that with aspirin (see Figure 8).

**Figure 8:** **Forest plots of the comparison of the Incidence of headache between cilostazol and aspirin group.** Heterogeneity test, chi-squarestatistic with degrees of freedom and *P* value; inconsistency among results, *I*^2^ test for overall effect, *Z* statistic with *P* value. CI, confidence interval; df, degrees of freedom; M-H, Mantel-Haenszel method.

## Discussion

Several antiplatelet agents, as suitable options for the secondary prevention drugs of ischemic stroke, are currently recommended by the American Heart Association and the American Stroke Association [19], such as aspirin, cilostazol, and clopidogrel [20,21].

Among these antiplatelet agents, aspirin is often prescribed as a mainstay agent for secondary stroke prevention because therapeutic monitoring is not required, it achieves a significant reduction in the absolute risk of acute ischemic and it is significantly lower in cost than all other antiplatelet agents [22]. Although aspirin has these advantages for secondary stroke prevention, in pooled analyses, it is reported [23] that its use is also associated with dosage-related gastrointestinal and intracranial hemorrhages. A significantly increase in the absolute risk of hemorrhagic stroke (+12 per 10,000 persons) has been reported, which translated to a relative risk increase of 84% with aspirin therapy [5]).

Recent clinical trial evidence suggests that cilostazol, a selective PDE3 inhibitor, may be a safer and more effective alternative than aspirin for secondary stroke prevention in Asian patients. Cilostazol’s utility is approved as a medication for ischemic stroke prevention by the Food and Drug Administration because it exerts antiplatelet and antithrombotic effects [24]. Studies reported that cilostazol reversibly inhibits the activation of PDE-3A, which is mainly distributed in platelets, heart muscle, and vascular smooth muscle. Cilostazol blocks platelet adenosine uptake and adenosine-induced platelet activation, to prevent platelet aggregation [25]. *In vitro* and *in vivo* data further demonstrate that cilostazol induces the expression of prostacyclin, which is the endothelium-derived antiplatelet compound, while aspirin allows for platelet aggregation through inhibition of COX and prostacyclin formation [26,27].

In contrast with aspirin for stroke prevention, which mainly has an antiplatelet effect, cilostazol also exerts vasodilatory effect and increases human carotid, cerebral, coronary, and dermal blood flow [27,28]. Emerging evidence suggests that cilostazol inhibits the PDE-3 enzyme in human smooth muscle cells, leading to effects on vasculature. These effects include inhibition of human smooth muscle proliferation by growth factors, reversion of intracranial atherosclerotic lesions, and improvements in cerebral blood flow [18,29]. Additionally, cilostazol increases levels of vascular endothelial growth factor, which serves to repair damaged vascular epithelium [27]. In our analysis, we collectively found a trend for the improvement of the efficacy of cilostazol over aspirin. Moreover, the combined properties of antiplatelet, antithrombotic, and effects on vasculature favorably contribute to the utility of cilostazol for stroke prevention [30].

Intracranial arterial stenosis is one of the most common causes of stroke worldwide and is associated with a high risk of recurrent stroke. Therefore, its prevention can reduce the risk of ischemic stroke. A randomized study of 135 patients with symptomatic intracranial arterial stenosis showed that treatment with cilostazol significantly reduced progression of the stenosis [31]. Moreover, cilostazol also significantly prevented progression of carotid artery intima-media thickness [32], which is an indicator of atherosclerosis and an established risk factor for stroke [33,34]. In our study, we found that cilostazol can significantly prevent progression of intracranial artery stenosis aggravation, as determined using MRA and TCD (MRA: combined OR 0.22, 95% CI (0.07, 0.68); TCD: combined OR 0.17, 95% CI (0.05, 0.51)).

It is well known that major bleeding is a main side effect of antiplatelet drugs, including aspirin. Some reported papers hint that there is evidence of fewer incidences of bleeding with cilostazol than with clopidogrel or aspirin [35], and our study confirmed those results (combined OR 0.38, 95% CI (0.24,0.60)). With respect to palpitation, the effect with cilostazol is almost as the same as that with aspirin, but cilostazol is associated with more minor adverse effects, such as gastrointestinal disorders (combined 1.23, 95% CI (1.04, 1.46)), dizziness (combined OR 1.44, 95% CI (1.15, 1.80)) and headaches (combined OR 1.78, 95% CI (1.52, 2.10)).

## Conclusion

Our meta-analysis of five RCTs investigated the safety and efficacy outcomes in ischemic stroke patients treated with cilostazol. The results showed that cilostazol might be a more effective and safer alternative to aspirin for patients with ischemic stroke. However, the number of surveys in the literature was limited and there might be a publication bias on application and interpretation. Additionally, recruited papers introduced little on allocation concealment, which is an important measure to ensure the quality of RCTs. Besides, there are few RCT studies focused on the effect of cilostazol on intracranial arterial stenosis and increased intima-media thicknessin patients with ischemic stroke. Further trials should examine the safety and efficacy of cilostazol in larger cohorts of patients and in comparison with other drugs currently used in secondary stroke prevention.

## Abbreviations

CI: Confidence interval; df: Degrees of freedom; MRA: Magnetic resonance angiography; OR: Odds ratio; PDE3: Phosphodiesterase 3; RCT: Randomized controlled trial; TCD: Transcranial Doppler.

## Competing interests

The authors declare that they have no competing interests.

## Authors’ contributions

YNQ and QB conceived of the study, participated in its design and coordination, draft the manuscript participated in performed the statistical analysis. Both authors read and approved the final manuscript.
